# A Multiattention-Based Supervised Feature Selection Method for Multivariate Time Series

**DOI:** 10.1155/2021/6911192

**Published:** 2021-07-20

**Authors:** Li Cao, Yanting Chen, Zhiyang Zhang, Ning Gui

**Affiliations:** ^1^School of Information, Zhejiang Sci-Tech University, Hangzhou, China; ^2^School of Computer Science and Engineering, Central South University, Changsha, China

## Abstract

Feature selection is a known technique to preprocess the data before performing any data mining task. In multivariate time series (MTS) prediction, feature selection needs to find both the most related variables and their corresponding delays. Both aspects, to a certain extent, represent essential characteristics of system dynamics. However, the variable and delay selection for MTS is a challenging task when the system is nonlinear and noisy. In this paper, a multiattention-based supervised feature selection method is proposed. It translates the feature weight generation problem into a bidirectional attention generation problem with two parallel placed attention modules. The input 2D data are sliced into 1D data from two orthogonal directions, and each attention module generates attention weights from their respective dimensions. To facilitate the feature selection from the global perspective, we proposed a global weight generation method that calculates a dot product operation on the weight values of the two dimensions. To avoid the disturbance of attention weights due to noise and duplicated features, the final feature weight matrix is calculated based on the statistics of the entire training set. Experimental results show that this proposed method achieves the best performance on compared synthesized, small, medium, and practical industrial datasets, compared to several state-of-the-art baseline feature selection methods.

## 1. Introduction

With the development of IoT, more and more domains, e.g., social media and industries, have accumulated a large amount of high-dimensional data with temporal orders, so-called multivariate time series (MTS), which contain valuable information. MTS data containing a large number of features become more and more common in various applications, such as in biology [1], multimedia [2], social networks [3], energy [4], and industries [5, 6]. It has brought the curse of dimensionality and volume. Excessive numbers of features may greatly slow down the quality of the classifiers because irrelevant, redundant, and noninformative features are highly confusing in the learning process [7–9], while also increasing computational overhead. Thus, it is important to fully exploit the complex relationship from both temporal and variate dimensions and identify the most related variates and their most appropriate feature time stamps in respect to the supervision target.  Figure 1 shows the two different requirements for the feature selection in MTS. Finding those variables and their time lags is often of great importance in understanding physical/chemical models of the underlying systems.

Feature selection, by removing irrelevant and/or redundant features/variables, has been seen as an essential and crucial data preprocessing step for machine learning [10]. The supervised feature selection methods are normally categorized as the wrapper, filter, and embedded methods [7, 11]. Different feature selection algorithms exploit various types of criteria to define the relevance of features: similarity-based methods, e.g., SPEC [12] and Fisher's score [13], feature discriminative capability, e.g., ReliefF [14], information-theory based methods, e.g., mRmR [15], and statistics-based methods, e.g., *T*-score [16]. However, those feature selection methods normally suffer major problems: varying from computation scalability to stability. Recently, advances in tree-based solutions and deep learning-based feature selection and many deep learning-based feature selection methods have been proposed due to their effectiveness in processing massive data and rich modeling capability. Random Forest [17] calculates feature importance as the sum over number of splits. The extreme popularity of the gradient boosting methods also provides feature selection capabilities, e.g., the Xgboost [18] and LightGBM [19] calculate feature weight basically according to the numbers of times the feature is used. Li et al. [20] proposed a deep feature selection (DFS) by adding a sparse one-to-one linear layer. Roy et al. [21] use the activation potentials contributed by each of the individual input dimensions, as the metric for feature selection. Gui et al. [22] in their recent work use an attention mechanism for the general feature selection task as both attention mechanism and feature selection focus on selecting partial data from the high-dimensional dataset. However, those feature selection algorithms are designed for general data and treating the two-dimensional MTS data indiscriminately.

For MTS feature selection, partially due to its complexity, most research studies are optimized for certain domains, e.g., Wong et al. [23] propose the feature selection method based on the adaptive resonance theory for financial time series forecasting. Jimenez et al. [24] define a wrapper feature selection method based on multiobjective evolutionary algorithms for antibiotic resistance outbreak prediction. González-Vidal et al. [25] design a feature selection method for smart buildings. Those approaches generally limit in their respective domains and cannot easily be extended to other domains. Few feature selection methods have been proposed for general multivariate time series. Most of them have major limitations. For instance, Hido and Morimura [26] find the most appropriate time stamps for the whole set of variates. Some keep, e.g., Wong et al. 2012, the time windows invariant or the same for all features [23]. Sun et al. [27] used the Granger causality [28] discovery to identify causal features as well as the effective sliding window sizes in multivariate numerical time series. However, these approaches face the same limitation of Granger causality and may produce misleading results when the true relationship involves three or more variables and is incapable of the nonlinear causal relationship.

In this paper, a novel multiattention-based supervised feature selection (m-AFS) method is proposed to explicitly tackle the two different correlations. It translates the feature weight generation problem into a bidirectional attention generation problem with two parallel placed attention modules. The input 2D data are sliced into 1D data from two orthogonal directions, and each attention module generates attention weights from their respective dimensions.

The major contributions of our work are as listed as follows:

- An innovative biattention-based feature selection architecture is proposed to make dimension-specific feature selection methods with neural network-based solutions. This method proposes a systematic structure to generate two different feature weights from a different perspective with one coherent neural network structure. By reusing existing neural network computation advances, this architecture supports fast and scalable feature weight generation.
- Two different attention-based modules are proposed that formulate dimension-specific feature weight generation problems into attention-based attention weight generation problems: attention over time (AoT) and attention over variates (AoV). Those two modules are designed according to the different characteristics of two-dimensional features.
- A feature weight generation mechanism is proposed to generate a final feature weight matrix to unify two different feature weights across two dimensions with simple dot product operation. As the attention weight might have a huge disturbance during the training, the final feature weight matrix is calculated based on the statistics of the entire training set.

A set of experiments are designed on a set of datasets including both regression and classification problems. The highest predicting and classification accuracy, compared with existing popularly used baseline algorithms, has been observed on all tested datasets. To the best of our knowledge, m-AFS is the first attention-based neural network solution for MTS feature selection tasks.

## 2. Multiattention-Based Feature Selection

In this section, the overall architecture of m-AFS is illustrated and analyzed. Then, the major components of this architecture are illustrated.

### 2.1. Notation

For the clarity of symbol usage, this paper presents matrices as a bold uppercase character (e.g., A), vectors as a bold lowercase (e.g., a), and normal lowercase character for numerical values (e.g., a). For instance, a time series is a series of observations, *x*_*i*_(*t*);  *i*=1,2,…, *m*;  *t*=1,2,…, *d*, which is made sequentially through time, where *i* denotes the index of the measurements made at each time step *t* and *t* denotes the index of the time. Matrix *X*={*x*_*i*_(*t*_*k*_)*|i*=1,2,…, *m*; *k*=1,…, *d*} is used to indicate the feature selection space with *n* features and *d* time points before time *t*. Here, *d* represents the maximum time interval in respect to the current time *t*. For the feature selection task, our goal is to find the appropriate feature and time step with respect to the output *y*(*t*). Here, *y*(*t*) presents the value for the label at time point *t*. When *n* is equal to or greater than 2, it is called MTS.

### 2.2. Architecture

As discussed in Introduction, for MTS data, two different feature selection dimensions coexist: time dimension selection and variate dimension selection. Those two dimensions have respective characteristics and have to be handled differently. In the time dimension, the sequence of a single feature's correlation with the target at different time steps generally is of close characteristics: (1) same unit: the unit of value is uniform for the same feature; (2) continuity in values: the values in time sequence are generally continuous. Normally, the smaller the time interval, the smaller the difference between the front and back of the sequence of features. However, in the variate dimension, different features are heterogeneous in most cases. Therefore, the ways in which features are correlated with the label normally are quite different.

Similar to the embedded feature selection methods, m-AFS generates feature weight during a learning process. As shown in Figure 2, m-AFS consists of three connected modules, namely, the AoT module, the AoV module, and the learning module. The AoT and AoV modules are parallel arranged in the upper of m-AFS. AoT is responsible for computing the time dimensional weights with transformed one-dimensional data instead of the original data. Each variate has an AoT module and a set of attention weights *a*_*T*_^*i*^ is generated. Similarly, the AoV takes all variates at the same time step as its inputs and tries to find the correlation between variates and label. The two attention modules are placed in parallel to avoid convergence problem which exists in the sequential structure. The mutual influence between two modules hampers the learning module. The learning module aims to find the optimal correlation between the weighted features and the supervision target by solving the optimization problem. It connects the supervision target and features by the backpropagation mechanism and continuously corrects the feature weights during the training process. The AoT, AoV, and the learning module build the correlation that best describes the degree of relevance of the target and features together.

As shown in Figure 2, m-AFS is a loosely coupled and stacked structure. Thus, it is quite similar to extend the feature selection to data with more dimensions, e.g., temporal, spatial, and variable dimensions. Furthermore, the learning module can also be customized according to specific learning tasks, e.g., CNN or RNN.

### 2.3. Design of the Attention Module

The AoV unit, as shown in Figure 3, slices the sample along the time dimension and uses the variate vector on a single time step *t*_*j*_={*x*_1_(*j*), *x*_2_(*j*),…, *x*_*m*_(*j*)} as input. Firstly, a dense layer (denoted as *E*) is used to extract the intrinsic relationship to eliminate certain noise or outliers. The introduced dense network *E* compresses the original feature domain into a vector with a smaller size (adjustable according to specific problems), while keeping the major part of the information. As the size of *E* is normally much smaller than the size of variables, certain redundant variables will be discarded during this process.

Secondly, by using the extracted *E* as input, each *U* is assigned with a shallow neural network corresponding to the number of variables. The output of *U* represents the *j*th time step's variable attention distribution. To widen the difference between variables and avoid to take an effect on the time dimension, the softmax activation is used and the selection possibility of feature *j*, *p*^*j*^ is calculated with equation (1) and the output *a*_*V*_^*j*^ is calculated with (2):

(1) $$\begin{array}{c} p^{j}=w_{p}^{j}t_{j}+b_{p}^{j}, \end{array}$$

(2) $$\begin{array}{c} a_{V}^{j}=\text{softmax}\left(\tanh\left(w_{n}^{j}p^{j}+b_{n}^{j}\right)\right). \end{array}$$

For each input *X* with *m* feature and *n* time steps, the AoV modules generate *n* different attention vectors *a*_*V*_^*j*^ for different time stamps *j*. Thus, it creates a weight matrix *A*_*V*_={*a*_*V*_^*j*^*|j*=1,2,…, *d*}. Note that the parameters of AoV and AoT modules are summarized as *θ*_*a*_.

While the AoV unit calculates the variable attention, the AoT unit integrates the input information of all moments in the form of soft attention. It uses the time step vector of a single variable *x*_*i*_={*x*_*i*_(1), *x*_*i*_(2),…, *x*_*i*_(*d*)} as input and calculates the *i*th variable's corresponding attention vector *a*_*T*_^*i*^*|i*=1,2,…, *m* and matrix *A*_*T*_=*a*_*T*_^*i*^*|i*=1,2,…, *m* with a series of transformations which are similar to the AoV unit. For each variable, one AoT is used.

This design has two major functions: (1) the separation of two dimensions avoids mutual influence and accelerates convergence and (2) each component *a*_*T*_^*i*^ and *a*_*V*_^*j*^ in the interval (0,1) can force many feature coefficients to be small, or exactly zero to facilitate feature selection. Attention here is similar to some sparse regularization terms used in many sparse-learning-based feature selection methods.

### 2.4. Learning Module

The feature weights generated from m-AFS are from AoT and AoV, respectively. Therefore, it is important to merge the two sets of weights to facilitate global feature selection. Two dimensions of the original data have their different characteristics and cannot directly be used for selection. But after the transformations of the attention module, weights of both dimensions are unified within [0,1] and can be directly used to identify the importance of variables. Here, we contact the two attention weight matrices *A*_*V*_ and *A*_*T*_ by a pairwise multiplication operation ⊙ and the global dimension attention weight is as follows:

(3) $$\begin{array}{c} A=A_{V}⊙A_{T}. \end{array}$$

The 2D weighted inputs of the learning module *G* can be accessed by the following equation:

(4) $$\begin{array}{c} G=A⊙X. \end{array}$$

*A* is constantly adjusted during the learning process with backpropagation by solving the objection function as follows:

(5) $$\begin{array}{c} \underset{A}{\arg\;\min}ℒ\left[f_{\theta_{l}}\left(A⊙X\right)-Y\right]+\lambda R\left(\theta \right), \end{array}$$

where *θ*=〈*θ*_*a*_, *θ*_*l*_〉 and *R*(·) is often an *L*2-norm that helps to speed up the optimization process and prevent overfitting. Here, *λ* controls the strength of regularization. The loss function depends on the type of prediction task. For the classification tasks, the cross-entropy loss functions are usually used. For regression tasks, the mean absolute error (MAE) is normally used. Note that *f*_*θ*_*l*__(·) is a neural network with parameters *θ*_*l*_.

For a specific learning problem, m-AFS can use a network structure that best fits the particular task. For general value-based regression and classification tasks, we adopt the fully connected network for task learning. Other structures, e.g., LSTM and CNN, are also adopted.

### 2.5. Feature Score Generation

Considering the much larger amount of data and limited computing resources in the real scenario, as well as the risk of trapping into local optimum, the training of network is processed in batch. This limits us to getting global attention weights of only one batch inputted, resulting in degraded performance. To have a better understanding of the attention distribution, we use the trained model to evaluate the whole dataset, get each sample's global weight *w*_*s*_, and calculate the statistical feature score using the following equation:

(6) $$\begin{array}{c} F=\frac{\sum_{i=1}^{D}A_{i}}{D}, \end{array}$$

where *D* is the size of the dataset and *A*_*i*_ is the attention matrix generated by the trained model for the sample *i*. The average weight matrix *F* across the whole sample is used as the basis for the feature selection.

## 3. Results

In this section, we will conduct experiments to answer the following research questions:

- *Q*1: Does the selection achieve good accuracy or a small error in those datasets?
- *Q*2: Does it capable to select the most appropriate features from both the temporal and variate dimensions?

In the following section, we introduce the basic experiment settings and the comparisons of different methods on both synthetic and real-world datasets.

### 3.1. Experiment Settings

This section is divided into two main experiments. The first experiment verifies the feasibility of m-AFS on a synthetic data. Then, experiments on several real-world datasets from the UCI Machine Learning Data Repository are conducted.

#### 3.1.1. Evaluation Setting

The ratio of training data to test data is 8 : 2. m-AFS adopts the normalization method introduced in Section 2.5 to generate global feature weight from the weights of variable and the temporal dimensions. Other feature selection methods do not have the concept of hierarchically generating weights. Thus, other baseline algorithms select feature directly via their feature weights across all features.

#### 3.1.2. Baselines

The implementation of the feature selection methods compared in this experiment is from the open-source library [7] (https://github.com/jundongl/scikit-feature). This experiment compares the m-AFS with the following representative methods:

  Similarity-based methods: Fisher's score [29] and ReliefF [30] select features by finding the near-hit and near-miss instances using the l1-norm: FS_l21 (feature selection with l2, 1-norm) [31]
  Embedded method: RF (Random Forest) is a tree-based feature selection method provided by scikit-learn package

#### 3.1.3. Predictive Model Settings

The RF (Random Forest) is used as the classifier for the experiments to avoid using the same methods for feature selection and testing. Other classifiers are also tested, e.g., support vector machine (SVM) is too slow to be used in the large dataset, and KNN is also much slower than RF and displays no significant advantages over RF in most of the tested datasets. Since the feature subsets selected by different feature selection methods are different, it is not appropriate to use the same hyperparameters for prediction. Therefore, we use the grid search to find the optimal parameters for the prediction model and use these parameters to set the model and then test the prediction accuracy on the reconstructed feature set. For the regression tasks, the mean absolute error (MAE) is adopted while the percentage of classification accuracy is used for classification tasks.

Model parameters are initialized with the truncated normal distribution with a mean of 0 and a standard deviation of 0.1. The model is optimized by Adam. The batch size is set according to the size of samples, 100 for small datasets and 1000 for MNIST and noisy MNIST. The learning rate is the default value of Adam optimizer in Keras framework (0.002). Here, all trainable parameters are constrained by *L*2 regularization. The network setting of AoT is one hidden layer and AoV is with two hidden layers: the first layer *E* with 32 units and the second layer *U* with the length of time steps and the number of the variables, respectively. The *E* layer is with 512 units. As the structure is loosely coupled, the learning module can be easily replaced. The max training epoch is set at 100 and early stopping is adopted to avoid overfitting.

### 3.2. Experiments on the Synthetic Data

In order to verify whether m-ATP can accurately identify the related features, we performed feature selection in a synthesized nonlinear system with known dynamics. There are six variables that are uniformly random distributed. The output *y* is generated with the following function:

(7) $$\begin{array}{c} Y=X_{1}\left(t-1\right)*X_{2}\left(t-2\right)+X_{3}\left(t-5\right)+X_{4}\left(t-1\right)+X_{4}\left(t-4\right)+\\ X_{4}\left(t-5\right)+X_{4}\left(t-7\right)+X_{4}\left(t-8\right)+\sigma \left(0,0.1\right), \end{array}$$

where *x*1 ∈ [2,5], *x*2 ∈ [10,30], *x*3 ∈ [5,10], *x*4 ∈ [30,70], *x*5 ∈ [100,200], *x*6 ∈ [65,85], and uniformly distributed. As can be seen from this equation, only *x*1∼*x*4 variates are related to *y* at certain time stamps. At the same time, in order to simulate the noisy environment, Gaussian white noise *σ*(0,0.1) is added. The total number of samples of the simulation dataset generated according to the above principles is 5000. Here, *T* is set to 10, and the total number of samples becomes 4991.

We tested various feature selection algorithms on the datasets. Here, the major focus is to check whether those algorithms can effectively identify the correct time stamps. Thus, the feature weights generated by different methods are illustrated in Figure 4. Note that as other methods generate weight in ranges other than [0,1], in order to have straightforward comparisons, those weights are normalized to the same range. Of course, the order of feature weights for feature selection is kept unchanged. The darker the feature, the more likely it should be chosen. This figure clearly shows that m-AFS can correctly find all the most relevant time stamps. In contrast, none of the other methods can correctly identify both variates and time stamps, or even some of them. For instance, although RF achieves very sparse feature weight distribution, this distribution deviates significantly from the real system dynamics. Thus, their results might give misguidance towards the system's characteristics.

### 3.3. Experiments on Real-World Datasets

To further demonstrate the effectiveness of m-AFS in real-world cases, we conducted experiments in six publicly available time series datasets from UCI (https://archive.ics.uci.edu/ml/index.php), including three regression datasets and three classification datasets. Details about the dataset are shown in Table 1. The size of the data is calculated with the product of sample instances, maximum time window, and the number of variates to represent how many inputs are needed to be calculated.

Table 2 shows the partial experiments results on the six different MTS datasets with different percentages of selected features. Due to the fact that MTS data normally have strong autocorrelation in the temporal dimension, maximum 15% of features are selected.

Table 2 shows that m-AFS and RF achieve the best performance on almost all the datasets and normally have big performance advantage over the other methods. RF leads with small percentage over m-AFS in the top 5% range and m-AFS ranks first in most top 10% features. However, their performances are quite close. It shows that both methods can identify the most influential factors for the prediction. Other methods, e.g., the LS_121 have rather unstable performance in different datasets. LS_121 ranks first in the OD dataset while it ranks last in the EEG dataset. Both datasets are the classification task. We also notice that more selected features normally yield little improvement towards the final results. And in the bigger range of top *K*, similar results are observed.

Here, the Random Forest algorithm is chosen also as the classifier for prediction and classification due to its performance and accuracy. We have to admit that this choice gives RF some advantages over the other methods. However, SVM is too slow to finish those tasks and KNN displays not so well accuracy in those tasks.

### 3.4. Interpretability

For many mission-critical domains, it is important that the generated feature weights have good interpretability and represent real system dynamics. Partial feature weights from the best two methods: m-AFS and RF for *x*2, *x*3, and *x*4 of the SRU dataset are shown in Figure 5. It clearly shows that m-AFS generates more smooth feature weights and clearly identifies the system lags for variates *x*2 (around 5 7), *x*3 (around 14), and *x*4 (around 8 10). This result is quite close to the results deduced by domain expert supported with domain-specific data mining solutions [32]. Their conclusion is *x*2 (6), *x*3 (14), and *x*4 (10). However, results from RF hardly demonstrate this conclusion although it has the best performance in SRU.

These results also show the possibility that the global weight generation methods proposed have room for improvements. How to generate global consistent weights to facilitate the feature selection with two different dimension-specific weights still needs further investigations.

### 3.5. Computational Complexity

In Table 3, the computation overheads of different feature selection methods are illustrated. Note that AFS intentionally only uses the CPU rather than the GPU as the calculation devices to make a fair comparison. Theoretically, it can execute 3∼9 times faster on the GPU.

The overhead is measured with the execution time for the feature weight generation process. Results show that AFS has moderate computation complexity. For the training with 1000 steps, it takes about 10 s to 173 s for the feature weight generation. Its execution time increases almost linearly as the size of data increases. In contrast, Fisher's score and ReliefF suffer the high and unstable computation cost. Their calculation time does not increase exactly with the increase in data volume.

### 3.6. Discussions

#### 3.6.1. Possible Applications

Obtaining the most relevant features of the target system and the time node with the greatest impact is essential for the modeling of any sequential system. As machine learning is more and more applied to the modeling of time series systems, the accuracy of the model is getting higher and higher, and the required parameters are becoming more and more complicated. The improvement of the accuracy of the model is of course very important, but the increase in the complexity of the model leads to a decrease in the intelligibility and robustness of the model. For many application scenarios that require high model availability and robustness, such as modeling of industrial systems, the existing deep learning models often cannot meet the modeling requirements of intelligibility and robustness. In our work, by identifying the most relevant features, the most relevant time delays, and the important system parameters and through the actual industrial data, the delay calculation of this SRU dataset is consistent with the actual physical model, which effectively illustrates that this work plays an important role in the modeling of understandable industrial systems.

#### 3.6.2. Current Limitations

The current major limitation is in the difference of feature weight evaluation. Traditional feature selection solutions calculate the feature weights and select the most influential features from the global perspective. In contrast, m-AFS calculates the feature weight from two different dimensions. Although our solution provides better interpretability, it introduces complexities in evaluating their contributions in the global aspect. And we need to balance the attention weight from multiple dimensions as proposed in Section 2.5. We are working on a more effective solution to condense weights from multiple dimensions.

## 4. Conclusion

In this paper, a novel multiattention-based feature selection architecture is introduced for the supervised feature selection for MTS data. In this architecture, two different attention mechanisms are designed to make the temporal and variable selection according to different feature selection patterns. Specifically, for the temporal dimension, the feature weight problem is formulated into a weighted average problem. For the variate dimension, the variate selection problem is transformed into a binary classification problem for each variate. This architecture is designed to be easily stackable so it is possible to be extended to data with more than two dimensions. Experiment results show that m-AFS can achieve the best feature selection accuracy on most tested different datasets, compared with three off-the-shelf and widely used baselines.

In future work, we aim to develop more domain-optimized solutions for data with more than 3 dimensions. We are also working on the data-driven physical dynamics model reconstruction to enhance the model interpretability.

## Figures and Tables

**Figure 1:** Two-dimensional feature selection in MTS: temporal feature selection and variate selection, only partial variates and certain time lags of those variates relevant towards the label *y*.

**Figure 2:** Conceptual structure of m-AFS.

**Figure 3:** Attention structure for temporal dimension.

**Figure 4:** Feature weight distribution in the synthetic data. (a) m-AFS feature weight; (b) trace ratio; (c) RF; (d) ReliefF.

**Figure 5:** Feature weight distribution in the SRU dataset.

**Table 1:** Dataset information.

Dataset	Type	Var. no.	Win. size	Train/test	Size (million)
DC	*R*	7	20	1900/475	0.266
SRU	*R*	5	15	8053/2014	0.603
AEP	*R*	27	20	15772/3944	8.516
EEG	*C*	14	20	11968/2993	3.351
OD	*C*	5	20	6499/1625	0.650
WFRN	*C*	24	20	4349/1088	2.328

**Table 2:** Regression and classification accuracy with different percentages of selected features with the RF classifier.

	SRU (10^−2^)	DC (10^−2^)	AEP (10^−2^)	EEG (%)	OD (%)	WFRN (%)
Top 5% of selected features						
m-AFS	1.65	6.55	**3.09**	**89.98**	95.38	92.74
Fisher 's score	2.63	11.24	3.72	81.35	98.52	93.47
ReliefF	2.74	9.39	5.53	70.09	97.48	94.30
Trace	2.80	5.94	4.05	68.09	84.74	90.71
LS_l21	1.86	6.81	3.36	63.81	**99.01**	92.46
RF	**1.40**	**5.37**	3.29	82.15	98.58	**98.34**

Top 10% of selected features						
m-AFS	1.3	**3.18**	**3.22**	**95.16**	**99.26**	95.96
Fisher 's score	2.55	7.31	3.38	85.63	98.65	96.04
ReliefF	2.52	7.73	5.29	76.54	98.46	95.31
Trace	2.58	5.62	3.44	75.67	86.77	92.09
LS_l21	1.57	5.24	3.23	67.65	98.52	93.29
RF	**1.10**	3.88	3.61	85.36	99.20	**98.07**

Top 15% of selected features						
m-AFS	0.99	**2.80**	3.27	**96.26**	99.26	95.96
Fisher 's score	2.52	7.03	3.30	89.31	98.71	96.87
ReliefF	2.51	6.14	4.73	82.73	98.77	95.59
Trace	2.54	5.40	**3.15**	79.89	86.95	92.56
LS_l21	1.50	4.56	3.20	75.01	98.52	93.38
RF	**0.96**	2.81	3.60	86.97	**99.32**	**98.07**

**Table 3:** Comparisons of the computation overhead (in seconds).

Meth. dataset	DC	SRU	EEG	AEP	OD	WFRN
m-AFS	10	52	101	173	44	60
Fisher's score	16	1511	68	128	21	5.6
ReliefF	633	45594	412	2707	72	45
Trace ratio	1.3	30	95	185	19.2	10
LS_L21	1	1.4	12	20	3.5	3.3
RF	3	9	33	124	1.5	7.8

## Data Availability

All data can be found at https://archive.ics.uci.edu/ml/index.php.

## Abbreviations

MTS: Multivariate time series
m-AFS: Multiattention-based supervised feature selection
AoT: Attention over time
AoV: Attention over variates
Conv: Convolution
FC: Fully connected.
